The article "Clinical Value of Coagulation Index Changes in Early Diagnosis and Nursing Intervention for PICC-Related Venous Thrombosis in Tumor Patients" was published in 2022. Journal: Contrast Media Mol Imaging.

# Clinical Value of Coagulation Index Changes in Early Diagnosis and Nursing Intervention for PICC-Related Venous Thrombosis in Tumor Patients

**DOI:** 10.1155/2022/7579225

**Published:** 2022-08-13

**Authors:** Meihua Gai, Wenjuan He

**Affiliations:** ^1^Center for Rehabilitation Medicine, Rehabilitation & Sports Medicine Research Institute of Zhejiang Province, Nursing Department, Department of Rehabilitation Medicine, Zhejiang Provincial People's Hospital (Affiliated People's Hospital Hangzhou Medical College), Hangzhou, Zhejiang, China; ^2^Emergency and Critical Care Center, Nursing Department, Intensive Care Unit, Zhejiang Provincial People's Hospital (Affiliated People's Hospital Hangzhou Medical College), Hangzhou, Zhejiang, China

## Abstract

**Purpose:**

To explore the clinical value of coagulation index changes in early diagnosis and nursing intervention for PICC-related venous thrombosis in tumor patients. *Patients and Methods*. A total of 170 tumor patients hospitalized for the first time with catheterization were enrolled from February 2018 to June 2022. According to the diagnostic criteria of venous thromboembolism, high-risk patients with venous thrombosis within 13 days after catheterization were enrolled in the observation group, and those without thromboembolism were enrolled in the control group. Venous blood was taken from all patients on days 1, 5, 9, and 13 after catheterization to measure the change trend of coagulation indexes of patients and to compare the difference of coagulation indexes between the observation group and the control group.

**Results:**

PT values of all patients were within the normal reference range at days 1, 5, 9, and 13 after catheterization. Compared with the control group, the observation group was significantly reduced on days 5, 9, and 13 after catheterization (*P* < 0.05), and continued to decrease with the prolonging of time(*P* < 0.05). After catheterization, the values of all patients at each time point were lower than the normal reference range. Compared with the control group, the values of tumor patients in the observation group were significantly decreased on days 5, 9, and 13 (*P* < 0.05) and continued to decrease at each time point (*P* < 0.05). DD values in the observation group were all higher than the normal reference range on days 1, 5, 9, and 13 after catheterization. Compared with the control group, DD values in the observation group were significantly higher on days 1, 5, 9, and 13 after catheterization (*P* < 0.05).

**Conclusion:**

PT and APTT continued to decrease after catheterization, and DD kept fluctuating at a high level, highly suggesting the possibility of venous thrombosis. The nursing staff should keep high vigilance and give appropriate nursing intervention.

## 1. Introduction

Peripherally inserted central catheter (PICC) is an intravenous route that can be used for prolonged administration, such as long-term chemotherapy, long-term antibiotic therapy, or complete parenteral nutrition. Since it was first used in 1975, it has replaced high-infection methods such as subclavian vein, jugular vein, and thigh vein. The PICC is inserted from the superficial vein of the elbow, and the catheter tip is located in the deep vein of the central vein to avoid the direct contact between chemotherapy drugs and the arm vein and reduce the stimulation of drugs on the blood vessels, so it can effectively protect the upper limb vein. Due to its rapid administration ability and relatively low incidence of complications and infection rates, catheterization has been widely used in the department of anesthesiology, ICU, emergency department, medical oncology, and other clinical departments. PICC is a commonly used method for nutrient intravenous delivery, tumor chemotherapy, and drug delivery and has been widely used for tumor patients in clinical treatment [1–3]. PICC can be implemented bedside operation, contributing to the infusion of liquid medicine through the blood vessels of the arm directly to the heart vessels, delivering necessary nutrient solution and reducing the pain of patients repeatedly puncture [4–6]. In practical application, PICC causes multiple types of complications such as catheter blockage, leakage, catheter ectopic, catheter-related infection, and venous thrombosis [7–12]. Among these complications, PICC-related venous thrombosis is a common complication in tumor patients, which not only increases the number of unplanned extubation but also leads to pulmonary embolism, seriously threatening the life safety of tumor patients [13–18]. Therefore, finding a reliable biomarker of early diagnosis for PICC-related venous thrombosis is of great importance, which facilitates early diagnosis and intervention of serious consequences. This study investigated the value of coagulation index changes in the early diagnosis of deep vein thrombosis for patients with malignant tumor after PICC catheterization.

## 2. Materials and Methods

### 2.1. Participant's Enrollment

A total of 170 patients with malignant tumor who received PICC catheterization in our hospital were selected. The inclusion criteria were as follows: (a) malignant tumor patients with PICC catheterization; (b) complete clinical data; (c) patients who underwent Doppler ultrasonography after catheterization; and (d) patients and their families who actively cooperated with hospital. The exclusion criteria were as follows: (a) patients diagnosed with deep vein thrombosis before catheterization; (b) abnormal coagulation function; (c) incomplete clinical data; (d) patients with blood system diseases; and (e) patients who refused to cooperate with this research. This study has been approved by the medical Ethics Committee of the hospital, and written informed consent was obtained from the subjects. There were 76 cases of left arm catheterization and 94 cases of right arm catheterization. 112 patients were complicated with hypertension, 53 with diabetes, 119 with coronary heart disease, and 15 with chronic renal insufficiency. There were 110 smokers and 44 alcoholics.

### 2.2. Experiment Methods

PICC catheterization was conducted by professional nurses and some necessary information should be recorded immediately after the catheterization according to the survey data record form in appendix, which includes name, gender, age, admission number, placement way, color doppler flow imaging examination, complications when drawing tube. The venous blood of all tumor patients was taken on an empty stomach for examination after PICC catheterization. Indicators of coagulation function included prothrombin time (PT), activates partial thrombin time (APTT), fibrinogen (Fib), thrombin time (TT), D-dimer (DD), and blood platelet (PLT). All the diagnostic reagents and machine were from Starco Diagnostics (Tianjin) Co. LTD. Subjects were selected according to inclusion and exclusion criteria and were included in the control group or the experimental group according to the ultrasound examination results.

### 2.3. Statistical Analysis

SPSS 15.0 software was applied to conduct *χ*^2^ test and *T* test. *χ*^2^ test of two independent samples was used for counting data comparison, and *T* test of two independent samples was used for measurement data comparison.

## 3. Results

### 3.1. Basic Information

Table 1 shows the detailed information and data of deep vein thrombosis after PICC catheterization in patients with malignant tumor. Based on careful statistical analysis, no significant association was found in factors in history of smoking, history of alcoholism, arm of insertion, tumor location, or complicating disease. The only significant association was found in history of recent surgical trauma.

### 3.2. PT

PT fluctuated within the normal range on days 1, 5, 9, and 13 after catheterization in both experimental group and control group. There was no significant difference between the experimental group and the control group on the first day after catheterization, but PT significantly decreased in the experimental group compared with the control group on days 5, 9, and 13 after catheterization. In the control group, the PT value increased continuously after catheterization but remained within the normal reference range. In the experimental group, PT value continued to decrease after catheterization and was in a low position within the normal reference value range. The detailed information is shown in Figure 1.

### 3.3. APTT

The APTT values of the control group and experimental group on the 1st, 5th, 9th, and 13th days after catheterization were lower than the normal reference range. APTT values at each time point in the control group were not statistically significant. The APTT value of the experimental group continued to decrease, and there was no statistical significance in the APTT value on days 1, 5, and 9, while the APTT value decreased significantly on day 13th. On the first day after intubation, there was no statistical significance between the two groups, and on the fifth, ninth, and thirteenth days after intubation, the APTT vaule in the experimental group were significantly reduced compared with APTT value in the control group. The detailed information is shown in Figure 2.

### 3.4. DD

The values on the 5th, 9th, and 13th days after catheterization in the control group were higher than the normal reference values, while the values on the 1st, 5th, 9th, and 13th days after catheterization in the experimental group were higher than the normal reference values. Compared with the control group, the values of test group at each time point were significantly higher. There was no significant difference in DD values at each time point in the control group. In the experimental group, DD values of patients at the same time point had a large variation and fluctuated greatly among all time points, but there was no statistical significance in DD values between all time points. The detailed information is shown in Figure 3.

## 4. Discussion

Catheterization is an invasive operation. It stays in the blood vessel for a long time with various complications, high incidence of venous thrombosis, and is easy to cause fatal adverse reactions to patients. In order to reduce the incidence of thrombosis, we observed the changes of blood coagulation indexes in patients with catheterization, so as to provide a basis for the prevention of thromboembolism. In this study, we sought to identify factors closely related to venous thrombosis.. It has been reported that the values of tumor patients are within the normal range from before thoracotomy to the day after surgery,and there was no significant difference between preoperative and postoperative. [19–21]. However, in this study, we found that the values of PT and APTT of tumor patients in the experimental group continued to decrease after catheterization, and decreased to the lower limit of the normal reference range on the first day after catheterization, while the control group continued to increase within the normal range. Therefore, we believe that the continuous decrease after catheterization is highly indicative of the possibility of venous thrombosis.

In this study, the values of patients in the two groups were lower than the normal reference range during all the measurement time, which may be caused by the hypercoagulability of cancer patients. The value of patients in the control group fluctuated within a certain range, while the value of patients in the experimental group continued to decrease after catheterization. Therefore, we believe that the continuous decrease is highly suggestive of the possibility of venous thrombosis. The current study found higher rates of venous thrombosis in cancers of the gastrointestinal tract, ovarian, breast, and lung. We found that the DD value of the venous thrombosis group increased significantly on the 4th day after catheters, reached the peak on the 9th day, and continued to the 13th day. The level of the non-venous thrombosis group remained at the same level from the 1st day to the 13th day without significant change. Therefore, we believe that the continuous high DD level after catheterization indicates the possibility of venous thrombosis.

By collecting clinical data of tumor patients, this study made a comparative analysis of the changes of coagulation indicators after catheterization. The results showed that PT and APTT continued to decrease after catheterization, and DD kept fluctuating at a high level, highly suggesting the possibility of venous thrombosis. In order to reduce the occurrence of relevant venous thromboembolism, nursing staff should regularly check the coagulation indicators of patients, pay attention to its changing trend, and give targeted nursing measures to patients with high possibility of venous thromboembolism to prevent the occurrence of blood test. As far as we know, this is the first study which investigates the coagulation index changes in early diagnosis and nursing intervention for PICC-related venous thrombosis in tumor patients. We must acknowledge that current research has shortcomings. Because of simple laboratory conditions and limited funds, we have to admit the fact that the sample size of the current study is small. In future studies, we will include more patients and healthy people to make our results more reliable. Bioinformatics is a hotspot of current medical research, which contributes to the diagnosis, treatment, and prognosis of diseases [22–26]. In the future, we would combine bioinformatics analysis with PICC-related venous thrombosis, which may contribute to finding some useful biomarkers for disease diagnosis and prognosis.

## 5. Conclusions

PT and APTT continued to decrease after catheterization, and DD kept fluctuating at a high level, highly suggesting the possibility of venous thrombosis. The nursing staff should keep high vigilance and give appropriate nursing intervention.

## Figures and Tables

**Figure 1:** PT value on days 1, 5, 9, and 13 after PICC catheterization in both experimental group and control group. PICC, peripherally inserted central catheter.

**Figure 2:** APTT value on days 1, 5, 9, and 13 after PICC catheterization in both experimental group and control group. PICC, peripherally inserted central catheter.

**Figure 3:** DD value on days 1, 5, 9, and 13 after PICC catheterization in both experimental group and control group. PICC, peripherally inserted central catheter.

**Table 1:** Risk factors of deep vein thrombosis after indwelling PICC in patients with malignant tumor.

Parameters	Thrombus group (*n* = 110)	No thrombus group (*n* = 105)	*P*
Gender (*n*)			0.957
Male	22	92	
Female	11	45	

Age	52.70 ± 6.83	54.46 ± 7.40	0.207

Complicating disease			0.384
Diabetes (*n*)	21	91	
Hypertension (*n*)	11	42	
Coronary heart disease (*n*)	23	96	
Chronic renal insufficiency (*n* (%))	8	7	

History of smoking (*n*)			0.583
Yes	20	90	
No	13	47	

History of alcoholism (*n*)			0.839
Yes	9	35	
No	24	102	

History of recent surgical trauma			<0.001
Yes	9	1	
No	24	136	

Arm of insertion			0.804
Left arm	13	56	
Right arm	20	81	

Tumor location			0.477
Lung	6	30	
Stomach	12	33	
Liver	2	13	
Pancreas	5	12	
Colorectal	3	15	
Others	5	34	

## Data Availability

The data generated or analyzed during this study are included within the article.
